# The Protection for Personal Information Based on IoT Network Management and Data Sharing in Big Data Era

**DOI:** 10.1155/2022/5143396

**Published:** 2022-10-03

**Authors:** Yu Zhang, Hexiao Yin, Haoyun Dong

**Affiliations:** ^1^Criminal Justice School, Zhongnan University of Economics and Law, Wuhan 430073, China; ^2^School of Criminal Law, East China University of Political Science and Law, Shanghai 201620, China; ^3^School of Criminology, People's Public Security University of China, Beijing 100038, China

## Abstract

A few decades ago, the protection of personal information was basically in the state of none, with more and more problems due to personal information, such as the use of information to achieve fraud and the use of false information to publish bad information, causing great property losses to people's lives. People only began to have awareness of the protection of personal information. After this, the civil law protection of personal information in IoT management has been developed. In this paper, we present a comparative analysis of the application of data sharing and protection of personal information based on the Internet of Things (IoT) management, as well as the sharing mechanisms used in data information, the protection of information security, and the drawbacks, which explains the safety information analysis of personal information in the case of data sharing and the calculation method used by the IoT in data sharing. A comparative study found that on the basis of IoT management, the security and concealment of personal information have been improved by about 20%. In practical application, IoT also brings great convenience in information data sharing. It increases the efficiency of operation, reduces losses, and to a certain extent guarantees the security of people's individual information.

## 1. Introduction

With the establishment of the socialist system in China, the Chinese Communists have been relentlessly exploring the concept of economic and social development. Broadly speaking, the development philosophy of the CPC has undergone a transformation from economic development, which focuses on the growth of material wealth, to scientific development, and then to shared development. The concept of shared development is a new development concept introduced in response to the current real-life problems that need to be solved in China, reflecting the maturity and perfection of China's development concept, which is a new leap in China's development concept.

The degree of data sharing reflects the information construction status of a region or a country, and the more channels for data exchange, the higher the information construction status. To achieve data sharing, it should first created a unified set of rules for data exchange; there are standard data schemas, rules for creating data usage, and the scope of data usage, data transmission channels, etc., with standardized data patterns, so that users can use the prescribed data templates as much as possible. Secondly, it needs to create data usage rules and formulate corresponding data copyright protection, property rights protection regulations, and sign data usage agreements between relevant departments, so as to break through the information shelter between departments and regions and achieve true information interoperability.

Data is an asset of the enterprise, especially the enterprise through the use of data skills, which will allow the enterprise to find newer resources and capital in addition to traditional resources such as labor, goods, and property, which promotes the acceleration of the digital transformation of the enterprise. There are two points in helping enterprises digital transformation: one is a set of core applications within the enterprise, as a daily use operation; secondly, it has to effectively control and communicate with the outer customers and the merchants responsible for supply, using various skills to collect a large amount of data from the real world and analyze it to achieve information exchange and resource sharing. In this paper, it integrated the relevant social needs, conduct business interactions, and use data to confirm and make decisions to achieve data innovation for the One Economy template.

## 2. Related Work

Due to the changing sensitivities and guidelines described in technical regulations, there is a growing interest in environmental respect among consumers, regulators, and researchers. In this case, the European Union (EU) Directives 2002/96/EC and 2003/108/EC control the management of electrical and electronic equipment (WEEE). Gamberini, Gebennini, and Grassi proposed an innovative model for restoration network management, including a case study [1]. Much effort has been invested in building fast and adaptive management solutions to support self-help, self-managed networks. Considering the high complexity of today's network environment, with little credentials for its use in practical management solutions to achieve autonomous networks, Ayoubi et al. is the latest advancement in network softwareization and programmability through SDN and NFV [2]. Reconfigurable computing systems, intelligent automated systems, and cognitive and parallel programming systems that use very complex resources or patterns for communication require a well-structured and carefully implemented system. Modieginyane, Malekian, and Letswamotse implemented a software-oriented networking environment through a software-defined wireless sensor network (SDWSN) approach combined with discrete event, simulation (DES), and a highly scalable software-defined network (SDN) controller [3]. Mykhaylenko, Waehrens, and Slepniov discussed operational strategies related to the link between configuration and capabilities, especially with regard to internationalization [4]. Traditional server-client MCS architecture often suffers from high operational cost of centralized servers and poor scalability; Changkun proposed a new P2P-based MCS architecture in which sensing data are stored and processed in local user devices and shared among users in a P2P manner [5]. According to the current situation of the medical industry, it is difficult to validate, store, and synchronize clinical data, and there are many limitations for doctors and even researchers to access and share data. Xue, Fu, and Wang proposed a blockchain-based medical data sharing model with the advantages of decentralization, high security, collective maintenance, and tamper-proof [6]. Sanderson et al. assessed the willingness to participate in biobanks using different data sharing models, which showed that the willingness to participate in biobanks and other large research projects would be higher in more rigorous situations. He also assessed perceived benefits, concerns, and information needs [7].

## 3. Relationship between Domestic and International Data Sharing Profiles and Civil Law

### 3.1. Overview of Data Sharing at Home and Abroad

Data sharing is a cumbersome system that has generated questions and research that has spanned a wide range of countries; the questions are as follows: how to make the information shared by the data become concealed and authentic, how to ensure the authenticity of the information in the transmission of information, and how to ensure the safety of citizens' property has become a major issue of common concern in the world. From the status of global data sharing presentation, their research data deposition, preservation, and utilization are characterized by the following: research data deposition and management become current grassroots tasks, which are shared by various observatories supported by the government; data precipitation and inquiry programs are carried out simultaneously: data obtained from important scientific research projects supported by the state are provided for sharing after the personnel of the project have first thought about the research for a certain period of time, and a perfect specification template is developed to open a discussion on the concepts and methods of data sharing; the introduction of high technology has led to the use of data so that data resources can play their proper role in the advancement of science and social and economic development [8].

From the 1950s onwards, data sharing spread globally to accommodate the need for extensive research. Developed countries and many international teams are planning and acting to create systems for the management, research, and use of scientific data in order to stimulate progress in scientific research and major issues such as resources and the environment. It is mainly aimed at the questions brought by globalized data sharing and the drawbacks in data sharing, which is conducive to the development of data sharing by scientific and technological personnel to get more use; for example, in the late 1960s, ICSU created the Global Data Center (WDC), in which many countries participate and have grown to nearly 50 disciplinary centers, making information collection and storage exchange to global internationalization. It has become a national center for all disciplines and is responsible for the performance of the national data research and service center in this discipline, as well as a member of the International Data Core. The current direction of global development is to create a global and territorial data network and to build a part of the core data and information sites in other developing countries under the premise of observing data rules. It is mainly to collect and preserve information, to improve and strengthen the information network, to increase the volume, and to use the national data network board. After a period of struggle, the basic conditions for modern data sharing have been established in each sector, as well as the establishment of its own information network [9]. Through these information networks, a simple data analysis and application organization has gradually been formed, which provides favorable conditions for interscientific and interdisciplinary data sharing in China, and also gives a guarantee for the realization of the project. At the same time, with the help of the state, we have further created a system of application and data analysis that can provide services to domestic and foreign users, and we have shown our value in the development of scientific progress and international information interaction.

To further create a scientific data research system and sharing system and lay a solid theoretical foundation for development. Existing major systems mainly focus on adopting, integrating, using, and exchanging. Each system has a group of experienced technicians in data management and analysis. They have rich data management experience, and basic knowledge, and they all have computer instruments of different grades. Many systems come with client servers and LAN systems, and some have gone into the Internet [10]. For example, the public communication network and combined data exchange network of the Ministry of Posts and Telecommunications established by the state and the blueprint of the information superhighway proposed by the state have made remarkable contributions to the technology on data exchange, and sharing is shown in Figure 1.

### 3.2. Data Sharing and Personal Information Security Based on Civil Law

In the information age, network sharing is entering people's lives and their lifestyles are changing, and network instruments have greatly facilitated our lives and work [11]. However, there is a connection between network sharing and people's personal information. Using network technology, the dissemination of information is accelerated, fraud text messages on mobile phones, authorization information of various APPs, and various unknown phone calls received, and even some fraudulent text messages are directly related to our bank card information, and network data is slowly invading our personal information and threatening our information security. Because of the virtualization of the network, if the network information leakage caused by fraudulent behavior, it is difficult to trace the individual, but also for the network information, security brings a certain risk. In the context of data sharing, the sources of network information have obvious falsity and instability, and the content is relatively complex, with strong differentiation and diverse complexity [12]. Because of the special nature of data sharing, the structure and characteristics of data sharing are obviously different, and the data structure and data type are no longer enough to judge the desecurity factor compared to the traditional network, and the database of resources is not easy to find. In terms of traditional data content, most of them are read through intelligent analysis and judgment of the source of the information, and the relevant technical staff can obtain rational analysis of the resources from the network technology to determine the source of the data. The dissemination channels of network information are shown in Figure 2.

The difference between traditional network data and modern network data lies in whether the data are integrated and analyzed through new network data and new network structures to form a relatively large database [13]. The content of the database is relatively cumbersome, and the user orientation can be quite diverse. It is not necessarily necessary to extract data from the structured network, but it is possible to obtain information from the unstructured network. This has led to the development of the entire network data slowly to the terminal, into a whole network, in the era of data interoperability. It can be accessed through the data terminal to check the information needed; the scope of access is relatively wide; the normal basic information of citizens can be accessed. Through the investigation, it is found that half of the information in the database in the network structure is incomplete and lacks logic, and the rigor and integrity are not perfect, so it is easy to lead to information leakage, which is also its disadvantage. Because this information sharing is public and open, it also leads to the information of citizens being public and not confidential. In the case of data sharing, accidents caused by information leakage can easily occur, and the public property and health of citizens may be spied on by unscrupulous people, which can lead to crimes, and this is also a disadvantage in the case of data sharing [14].

### 3.3. Relationship between Network Data Security and Citizens' Personal Information Security

There are many ways of data sharing in the data system, such as electronic terminal mobile terminal, intelligent terminal, and other methods. Moreover, some of the contents on the network information belong to the real information, which makes it easy to have dangerous accidents. There are many unscrupulous people who steal personal information through the virtual environment of the network and provide false information to customers by providing services, which causes harm to citizens' money. In this way, the enterprise through the platform reserved telephone information and then communicate with customers; it is easy to lead many citizens to be cheated and seriously affect the green public network environment [15]. Unscrupulous elements mainly focus on fraudulent money; they also analyze and understand through the network information platform to determine the daily behavior of most citizens and places of access, as well as the consumption situation. Moreover, unscrupulous people can learn about users' daily behavior, consumption, geographic location, etc., through various channels. Therefore, for the sharing of network data and information leakage, there is a relatively large risk for users. Cyber crooks can use this information to process citizen data and then analyze it accurately, leading to the exposure of citizen information [16]. We also need to protect citizens' personal information according to the law, as shown in Figure 3.

### 3.4. Data Sharing and the Sharing Mechanism of Cloud Data

Under the premise of cloud computing, data information is widely used, and the capacity of data is gradually expanded to form decentralized storage. Cloud computing is scattered, malleable, and practical in analyzing data, all of which are outstandingly demonstrated in cost forecasting [17]. In the decentralized data system, the most prominent characteristic of it is to have data redundancy under regular circumstances. The problem of redundant data configuration in decentralized storage under cloud computing is of great significance to ensure the robustness of data and also forms a hot topic for deep investigation by related scientists at present. Previously focused on the problem of redundant data mass configuration for big data, it mostly using support vector machine algorithms as the main approach. This method specifies the fragmentation update factor and dynamic cost factor. Based on the selection of the minimum cost of data movement nodes, it uses parameter iteration to estimate the cost of segments from scratch to nodes and mostly uses dynamic class core allocation to classify big data. One of them is to categorize the redundant data in the decentralized storage of big data in cloud computing, and the other is to divide the redundant data paragraphs after classification. This improves the configuration accuracy and configuration efficiency of redundant data, which is then transformed into finding the best solution to the plane problem after the categorization operation in the data.

(1) $$\begin{array}{c} R\left(\beta \right)=\overset{p}{\underset{j=1}{\sum }}\beta_{j}-\frac{1}{2}\overset{p}{\underset{j,k=1}{\sum }}\beta_{j}\beta_{k}Z_{j}Z_{k}\left(y_{j}•y_{k}\right), \end{array}$$

where *R*(*β*) is the bilevel definition function, *y*_*j*_•*y*_*k*_ is the vector product, and *Z* is the categorical definition value; *Z*_*j*_ and *Z*_*k*_ are the categorical definition values of the two vectors *y*_*j*_*y*_*k*_, respectively; *β* is the proportional mechanism vector; and *β*_*j*_*β*_*k*_ denotes the proportional weights of the two vectors *y*_*j*_*y*_*k*_, respectively. *p* is the core maximum, and the following conditions must be observed for the plane to find the optimal solution.

(2) $$\begin{array}{c} \overset{p}{\underset{j=1}{\sum }}Z_{j}\beta_{j}=0, \end{array}$$

(3) $$\begin{array}{c} \beta_{j}\geq 0,j=1,2..,p. \end{array}$$

Assuming that the redundant data in the distributed storage of big data under cloud computing causes special nonlinear transformation, it is required to use the inner product *L* (*y*_*j*_ · *y*_*k*_) to replace the product in the optimal classification function; then, the optimal classification plane solution problem is transformed into the objective formula:

(4) $$\begin{array}{c} R\left(\beta \right)=\overset{p}{\underset{j=1}{\sum }}\beta_{j}-\frac{1}{2}\overset{p}{\underset{j,k=1}{\sum }}\beta_{j}\beta_{k}Z_{j}Z_{k}L\left(y_{j}\cdot y_{k}\right). \end{array}$$

Assuming that Formula (5) is the best categorization function of Formula (4), then:

(5) $$\begin{array}{c} g\left(y\right)=\mathrm{sgn}\left(\overset{p}{\underset{j=1}{\sum }}\beta_{j}Z_{j}L\left(y_{j}\cdot y_{k}\right)+c^{\prime }\right). \end{array}$$

In the formula, *g*(*y*) is the optimal classification function, and *c*^,^ is the type attribute. Through this function, redundant data paragraphs can be obtained. The optimal classification plane algorithm can classify two types with differences. However, the redundant data in the distributed storage of cloud computing big data belongs to multiple categories, so it is necessary to first convert the redundant data classification in the distributed storage of cloud computing big data into a variety of optimal classifications, and then solve them one by one, and finally obtain the classification results of redundant data in the distributed storage of big data under cloud computing. Currently, the two classifications are generally single-to-multiple or single-to-single classification [18]. Because the configuration of redundant data of big data under cloud computing is not small, and the special values of redundant data are too many, it is necessary to use a single-to-single classification method, to run the transformation measures of redundant data classification in the distributed storage of big data under cloud computing.  Figure 4 shows the flow chart of redundant data configuration for distributed storage of big data under cloud computing:

The above mainly solves the configuration process of a redundant data segment in the distributed storage of cloud computing big data, establishes configuration strategies and estimation criteria, and obtains the optimal redundant data configuration strategy. The cost formula is to combine the unified information of each item to estimate the communication value of redundant data. Its value formula is:

(6) $$\begin{array}{c} sum\cos t=g\left(y\right)\underset{F}{\sum }\cos t\left(F_{j}\right). \end{array}$$

In the formula, *sum*cos*t* represents the communication cost corresponding to the overall data configuration strategy, *g*(*y*) is the classification result of redundant data in the distributed storage of big data under cloud computing in the previous section, and cos*t*(*F*_*j*_) is the communication value corresponding to the configuration strategy in data paragraph *F*_*j*_.

(7) $$\begin{array}{c} \cos t\left(F_{j}\right)=T_{Q}\left(F_{j}\right)+T_{U}\left(F_{j}\right). \end{array}$$

*Q*, *U* in the formula represents the classification corresponding to the configuration strategy of different data paragraph *F*_*j*_, and the communication value is expressed by *T*_*Q*_*F*_*j*_, *T*_*U*_*F*_*j*_, and their calculation formulas are:

(8) $$\begin{array}{c} T_{Q}\left(F_{j}\right)=\underset{Q}{\sum }\underset{S_{k}}{\sum }delay{\left(S_{k},S_{c}\right)}_{\min}, \end{array}$$

(9) $$\begin{array}{c} T_{U}\left(F_{j}\right)=\underset{U}{\sum }\underset{S_{k}}{\sum }\left[\underset{S_{c}}{\sum }delay\left(S_{k},S_{c}\right)\right]. \end{array}$$

Among them, *S*_*k*_ is the site where things Q and U appear, and the storage section *F*_*j*_ is set to *S*_c_ in the configuration policy. If the configuration strategy has redundancy, *S*_c_ is changeable, and the corresponding value of *delay*(*S*_*k*_*S*_*c*_) is also changeable. In formula (7), *dalay*(*S*_*k*_*S*_*c*_)_min_ is the corresponding minimum value, and ∑_*S*_*c*__(*delay*(*S*_*k*_*S*_*c*_) is the algebraic sum of the values.

According to the above classification results and classification process, it is concluded that the redundant data configuration strategy implemented in this paper is as follows:

1. Set the evolution coefficient

According to the essential problem, reasonably set the evolution coefficient of redundant data given in advance; for example, *np*, *ng* represents the number of redundant data populations and the stop evolution coefficient, respectively.

(2) Encoded into a string of bits

The result of the problem, as the configuration of paragraph *F*_*j*_ in the data, is expressed in binary, assuming that *F*_*j*_ is classified as station *S*_*k*_, and the *k*th number in the structure is obtained. Suppose it is “1,” if the corresponding digital structure is not obtained in the structure, then it is “0.” It is calculated that there are (2^*m*^ − 1) kinds of corresponding structures in paragraph *F*_*j*_, and the estimated total value of string bits is cos*t*(*F*_*j*_), and the number of added data paragraphs is *q*. Then, in this overall structure, it can be turned into a *q*-row *m*-column table, a total of (2^m^ − 1) types, and each type has a different and special total communication value.

(3) Initialize the group

Due to the characteristics of the original group of *sumco* and efficiency redundant data, the breeding method is used in the redundant data allocation algorithm of the genetic algorithm to implement the originalization. In the first step, *np*0 individuals are randomly formed, and in the second step, *np* individuals with the smallest corresponding communication value are selected to form the original population. This method can ensure that the original internal individuals of redundant data reach a higher level.

(4) Calculate the individual fitness value

Formulas (7), (8), and (9) obtain the communication value corresponding to each individual in the redundant data group one by one, and the reciprocal of the value is the value of the individual's fitness.

(5) Selection processing

The redundant data allocation algorithm based on genetic algorithm combines the best storage and data selection to implement individual sampling selection processing. When the fitness of the best individual in the offspring is not as good as that of the parent, the best individual in the parent is used to replace the worst individual in the offspring to ensure the stability of the algorithm. In order to establish a relatively stable selection process and prevent a special individual from being excessive in the group, the fitness of individual individuals is judged to obtain a probability value to determine whether it can be run [19]. The careful steps are as follows: the data distribution of the obtained fitness in the computer data is sorted in order, and the amount of data is *np*; secondly, important parameters need to be set, *p*_0_ is 1/*np*, and then, the order of individuals is obtained according to the probability. Then, each individual serial number can be expressed as *j*_0_, with:

(10) $$\begin{array}{c} p_{j}=\frac{p_{0}{\left(1-p_{0}\right)}^{j-1}}{1-{\left(1-p_{0}\right)}^{np}}. \end{array}$$

(6) Interspersed processing

*GA*2 Using the single-point interleaving method under the general constant probability *p*_*c*_ can enhance the running probability of the algorithm.

(7) Alienation treatment

The lack of mature convergence is relatively common in genetic algorithms and belongs to a high probability event. In the previous genetic algorithm, the generally selected value is relatively small, and the probability of alienation is also reduced accordingly. If there is early convergence, it will be difficult to obtain the local optimal solution. In order to implement and automatically become multiple new individuals, the redundant data allocation algorithm of the genetic algorithm can quickly increase the complexity of the redundant data group and help the group to get rid of the premature convergence, so as to obtain the expected results. Using the method of alienation processing, it is possible to check whether the maximum fitness value and the average fitness meet the standard, and whether to converge, *f*_max_ < *f*_*vag*_. Assuming that the density factor is *t*, it represents the mean situation, between 0 and 1. If the value is close to the median, the probability of alienation will be too high. After reaching the numerical requirements, select a probability *p*_max_ that is 5 times greater than *p*_*m*_ from the numerical values and perform alienation processing. If not, the alienation process will be implemented according to the original probability of *p*_*m*_. If *p*_max_ increases, it can also indicate that the operation is stable, and an appropriate reduction in the convergence rate can be used. If *p*_max_ is 0.5, the system will convert to random query [20].

(8) Judging whether the stopping criterion is met

If evolutionary algebra *gen* is less than evolutionary algebra *ng*, the system will return to the previous step and re-selection. If *gen* is not less than *ng*, then get the last system data, then jump to the last step. The individual with the highest final fitness of the decoded data will finally obtain the optimal configuration method of data segment *F*_*j*_. Aiming at the problem of slow exercise rate of large-scale experimental samples, a center calculation method for the vertical bisector of the center line segment is proposed. According to the distance samples from each experimental data to the vertical bisector, save the samples to obtain a new training book. The new training book is used to replace the original training book, and SVM training is implemented to achieve the purpose of improvement [21]. In the support vector machine algorithm, different hyperplanes need to be solved for the classification and solution of the training book. In order to implement this operation, the planes are first normalized. Let *ζ* = 1, so that the closest vector samples satisfy the following conditions (equal when *ζ* = 1):

(11) $$\begin{array}{c} \left(\omega^{T}x^{*}\right)+b\geq +1,y=+1, \end{array}$$

(12) $$\begin{array}{c} \left(\omega^{T}x^{*}\right)+b\leq -1,y=-1, \end{array}$$

In the formula, *ω* is the data vector of the system plane, *b* is the numerical item of the rule function, *y* is the type sample item, and *x*^∗^ is the purpose support vector.

If the distance between the hyperplane and the target support vector is 1/‖*ω*‖, then the original problem can be transformed, so that the solution of *y* is a convex programming problem.

(13) $$\begin{array}{c} M\text{in}\Phi \left(\omega \right)=\frac{1}{2}{\left\|\omega \right\|}^{2}, \end{array}$$

(14) $$\begin{array}{c} s.t.y_{i}\left(\omega^{T}-b\right)-1\geq 0,i=1,2,\cdots \end{array}$$

Bring it in and get *W* = ∑_*i*=*Ω*_*SV*__*α*_*i*_^∗^*y*_*i*_*x*_*i*_. After judging the plane of vector *Ω*_*SV*_, it satisfies the system space of the vector in its interior, and after operation to Lagrange *α*_*i*_^∗^, the value of the support vector is not 0. By calculating the value of the purpose support vector, it is judged whether the available classification surface can be constructed [22]. After running the classification algorithm, classifying through the classification surface, and then substituting the formula into the above formula, the indicator function in the following formula can be obtained:

(15) $$\begin{array}{c} f\left(x\right)=\mathrm{sign}\left[\underset{i\in \Omega_{SV}}{\sum }y_{i}\alpha_{i}^{*}\left(x_{i},x\right)-b^{*}\right]. \end{array}$$

It can be seen that the training book of the support vector machine is only related to the support vector and has nothing to do with the nonsupport vector. The support vector is often at the edge of the sample, so the boundary vector can be extracted as a new training book for testing while ensuring the classification ability of the support vector machine, thereby improving the classification probability. To solve the “curse of dimensionality” problem, a new concept function kernel function is introduced. By solving the kernel function *K*(*x*_*i*_, *x*), the product of *x*_*i*_ and *x* in the actual problem of *wolfe* is replaced by *K*(*x*_*i*_, *x*). By introducing a new kernel function *K*(*x*_*i*_, *x*), the discriminant function can be:

(16) $$\begin{array}{c} f\left(x\right)=\mathrm{sign}\left[\underset{i\in \Omega_{SV}}{\sum }y_{i}K\left(x_{i},x\right)-b\right]. \end{array}$$

By introducing a kernel function, the original problem can be extended to a high-dimensional space by means of a product in the calculation process.

### 3.5. Disadvantages of Data Sharing

The disadvantages of data sharing include high difficulty in data control, instability of data storage parties, wide range of data sharing fields, and data security risks. Data sharing covers a wide range of people, and it controls a large number of people. Data sharing relies on the control of data. However, the instability of the data storage party increases the difficulty of data control and reduces the data ontology's ability to control data. In addition, data sharing has high technical requirements for data controllers; data controllers should have the capabilities of data storage, security assurance estimation, skill processing, etc.; and the data sharing ontology has certain verification tasks for information recipients to prevent data problems [23]. However, due to prescriptive financial considerations and lack of positive incentives, most data controllers often ignore data risks and share data. When the data is shared beyond the original amount of data storage, most of them are reluctant to obtain the approval of the data ontology again. The sharing of privacy policies on 100 platforms is shown in Figure 5:

Data sharing accelerates the generation of data rationality errors and data discrimination. Data is more rational, but data is not necessarily conclusive, and data discrimination caused by data errors is more difficult to change. Based on the judgment of “data portrait,” most of the enterprises will become the situation of big data killing, price financing contempt, and so on. Even when the relevant data of the data ontology has changed, the data portrait still exists, making it difficult to solve the “data problem.”

## 4. Comparative of IoT Management Based on Data Sharing

As information becomes more and more shared and simplified, we will gradually show some problems in the management of the Internet of Things, such as the risk of personal information leakage on the platform, the lack of concealment of the platform's own information, and the imperfect management of the Internet of Things. Personal information is no longer safe, which is also a concern for many people. In the case of data sharing, it is also necessary to strengthen the confidentiality and confidentiality of personal information. Under the same circumstances, whether the information of the Internet of Things is trustworthy, will it be more secretive and secure. The experimental comparison of this result is shown in Figure 6:

Through comparative research, it is found that in the management of the Internet of Things, the safety factor between groups and enterprises is higher, with an increase of about 20% year-on-year. In the case of data sharing, enterprises and the masses will become more secure between individuals, and you can rest assured that there will be a layer of protection in the transmission of information. At present, problems caused by personal information leakage are also generally increasing. Strengthening personal information and protecting oneself is also a major task of IoT information management.

The era of data sharing has indeed brought great convenience to people's lives, but it has also made a lot of information public. More and more people do not carry cash but pay through a treasure, a letter, etc. But it does not take into account why you need your location to turn on the phone's lighting or read your address book when you turn on the phone's radio. Many apps even automatically read your mobile phone information, positioning, etc., by default, which undoubtedly makes the information transparent. We have also become “transparent people,” and then, our own information is exposed on major data platforms, followed by telecommunication fraud, privacy invasion, telephone harassment, advertising push, etc. These leaked information, on average, everyone has four pieces of relevant information, which makes people shudder, and the economic losses caused by them are also immeasurable. A comparative analysis of this aspect and IoT management is made, as shown in Figure 7:

In contrast, IoT management reduces the incidence of accidents and minimizes economic losses. The economic loss from telecommunication fraud has been reduced by about 25%, the incidents of privacy violations have also been reduced by 15% in the same year, and the amount of harassment by phone and text messages has also been reduced by 20%. It is not difficult to see that the management of the Internet of Things does help a lot in information security, but there are still many that have not been completely eliminated. To reduce people's daily troubles at the social level, in the era of data sharing, we should not be greedy for petty cheap, do a good job of self-economic prevention awareness, learn more knowledge, and minimize unnecessary economic losses.

In modern transportation, there are many traffic incidents every day. In the case of data sharing, information communication can be used to solve problems in a timely and effective manner, which brings great convenience to the traffic police. From the integration of data, the information of the upper and lower departments can be effectively unified, and the information of the relationship layer is more closely connected. In the collection of resource information, various data can be submitted and judged at almost the same time, and the traffic police can handle it according to the current situation. To be fair, just and timely, the interoperability of the national traffic police network has strengthened the exchange of information and the handling of special matters, and the mutual sharing ability has been improved. As shown in Figure 8, the efficiency improvement of data sharing in transportation is compared.

Through data comparative analysis, it can be found that the data collection efficiency has increased from the previous 55% to 75%. In terms of information integration, it has increased from 67% to 88%, and the overall improvement is still very good, with an increase of about 20%, which reduces the time for information traffic and avoids long-term processing of special problems. The benefits brought by data sharing are still visible. Compared with the situation without sharing, the improvement will be greatly reduced.

Hospitals have a close relationship with people's daily life and play an extremely important role. However, the current medical situation is difficult to be reassuring, and there are often patients who cannot receive timely and effective treatment. The management of the hospital itself cannot keep up with the development of the times, nor can it meet the medical needs of people in the new era. With the continuous deepening of the application of Internet of Things technology in China's medical industry, scientific and intelligent management under computer control has been truly realized. As shown in Figure 9, IoT management allows hospitals to intelligently arrange numbers, establish a communication platform, and compare the optimized management brought by real-time monitoring of drugs and equipment IoT connections.

By comparison, it is found that patients need less time on intelligent scheduling, which is 33% less than before, which also shows that IoT management has indeed brought certain convenience to the hospital and greatly shortened the waiting time. The information exchange between patients has also become faster and more synchronized, and the efficiency has increased by about 43%. Hospitals can also carry out batching, special treatment for different groups of people; distinguish the situation; and make early judgments. For the hospital itself, the use of medical equipment can be accurately controlled, as well as the situation of drugs, can be known in advance. This saves the time for checking out materials and equipment and saves one-third of the previous time compared with the previous year, which greatly facilitates patients and medical staff.

## 5. Discussion

Data sharing has become an indispensable and important technology in today's society, and it has become a beacon for the development of the information age, guiding future generations. Every technology has its pros and cons. The main thing is to improve it slowly in application and improve it gradually in practical problems. In the management of the Internet of Things, it is necessary to continuously optimize the data processing in it. Analyzing the existing problems to reduce harm to citizens, reduce the spread and packaging of false information on the Internet, can strengthen network health management, so that future data sharing will always be at the forefront of technology. In this environment, people will become more and more secure, regain trust between people, and there will be no more online fraud what is believed this is that every citizen looks forward to most.

## 6. Conclusion

This paper mainly compares and analyzes personal information security issues in data sharing under Internet management and finds that data sharing has greatly facilitated people's lives and has a certain protective effect on citizens' information. However, there are also certain drawbacks. Technology is a double-edged sword, and it still depends on how people use it. At the same time, we must strengthen our own personal information protection and reduce unnecessary risks as much as possible. Strengthen your own understanding of the Internet of Things and data sharing, so as not to be addicted or fallen, but use it as a tool for learning and use, constantly improve the information of data sharing, and learn and progress.

## Figures and Tables

**Figure 1:** Framework diagram of IoT database.

**Figure 2:** The dissemination path of network information.

**Figure 3:** Protection of personal information according to law.

**Figure 4:** Flowchart of big data distributed storage redundant data configuration under cloud computing.

**Figure 5:** 100 platform privacy policy sharing and utilizing special authorization.

**Figure 6:** Personal information security comparison.

**Figure 7:** Comparison of economic losses under IoT management.

**Figure 8:** Comparison of efficiency improvement.

**Figure 9:** Comparison of management optimization of IoT in hospitals. (a) Original optimization management diagram. (b) Management diagram after IoT optimization.

## Data Availability

The data that support the findings of this study are available from the corresponding author upon reasonable request.
